# Application of Nursing Outcome-Oriented Integrated Zero-Defect Nursing Combined with Respiratory Function Training in Long-Term Bedridden Patients Undergoing Stroke

**DOI:** 10.1155/2022/4425680

**Published:** 2022-09-30

**Authors:** Shaona Xu, Yanan Yu, Hongling Liu, Weiwei Qiu, Yu Tang, Ying Liu

**Affiliations:** ^1^Department of Neurosurgery, Yantai Affiliated Hospital of Binzhou Medical University, Yantai, Shandong 264100, China; ^2^Department of Surgery of Thyroid Gland and Breast, Yantai Affiliated Hospital of Binzhou Medical University, Yantai, Shandong 264100, China; ^3^Department of Neurology, Yantai Affiliated Hospital of Binzhou Medical University, Yantai, Shandong 264100, China; ^4^College of Basic Medicine, Binzhou Medical University, Yantai, Shandong 264000, China

## Abstract

**Objective:**

To explore the application effect of nursing outcome-oriented integrated zero-defect nursing combined with respiratory function training in long-term bedridden patients with stroke.

**Methods:**

A total of 120 long-term bedridden patients with stroke were randomly divided into three groups: groups A, B, and C. Group A was given nursing outcome-oriented integrated zero-defect nursing combined with respiratory function training, group B was given nursing outcome-oriented integrated zero-defect nursing, and group C was given routine nursing. Rosenbek aspiration degree classification criteria were used to evaluate the incidence of aspiration; blood oxygen saturation, arterial oxygen partial pressure, and respiratory pressure were compared before and after the intervention. The swallowing function was evaluated by a water swallowing test (WST). The quality of life was assessed using the Generic Quality of Life Inventory-74 (GQOLI-74).

**Results:**

After treatment, the Rosenbek aspiration degree of groups A and B were better than those of group C (*P* < 0.05); the improvement degree of respiratory function indexes in group A was better than those in B and C, and the blood oxygen saturation and arterial blood oxygen partial pressure in group B were better than those in C (*P* < 0.05). The incidence of complications in groups A and B was lower than that in C, and complications in group A were lower than that in B (*P* < 0.05). After treatment, the scores of psychological function, social function, and material life status of the three groups were increased, and each score of groups A and B was higher than that of C, and each score of group A was higher than that of B (*P* < 0.05).

**Conclusion:**

Nursing outcome-oriented integrated zero-defect nursing combined with respiratory function training can effectively improve aspiration, respiratory function, swallowing function, complication rate, and quality of life in long-term bedridden patients with stroke.

## 1. Introduction

Stroke is a cerebrovascular disease caused by the blockage or rupture of cerebral blood vessels that prevent blood from flowing into the brain. It has the characteristics of high morbidity, high mortality, and high disability rate, which is a serious threat to the life and health of patients [1, 2]. 60% to 70% of strokes are ischemic strokes caused by internal carotid artery occlusion and stenosis. At present, most of the clinical treatment of strokes is thrombolytic and antiplatelet therapy. Some stroke patients can get out of danger in time after treatment. However, about 80% of patients may have different mental and limb dysfunction. Most of them have respiratory dysfunction, swallow dysfunction, and lung infection. Due to the lack of consciousness of stroke patients for a long time, the cough is weak and the ability to expel sputum is lost, which eventually leads to pulmonary infection [3–5]. Respiratory tract infection will lead to a continuous increase in the mortality rate of stroke patients, seriously affecting the rehabilitation of patients. High-quality nursing guided by nursing results can determine nursing objectives according to patients' clinical data, adopt targeted nursing methods to meet the needs of patients, and improve the situation of blind unified nursing in traditional nursing. Zero-defect nursing mode emphasizes general comprehensive nursing, which can effectively avoid adverse events and loopholes in nursing and improve patients' nursing satisfaction. The normal swallowing process includes respiratory tract protection and esophageal promotion, which can affect swallowing function.

In this study, the comprehensive zero-defect nursing combined with respiratory function training was conducted to long-term bedridden patients with stroke to explore its application effect.

## 2. Materials and Methods

### 2.1. General Information

120 patients with long-term bedridden stroke treated in our hospital from May 2020 to June 2022 were randomly divided into three groups: group A (*n* = 40), group B (*n* = 40), and group C (*n* = 40). In group A, there were 22 males and 18 females, aged 51–78 years, and the average age was 65.38 ± 5.99 years old; 15 cases of left hemiplegia, 19 cases of right hemiplegia, and 6 cases of bilateral hemiplegia; 12 cases of cerebral hemorrhage and 28 cases of cerebral infarction. There were 24 males and 16 females in group B, aged between 53 and 77 years old. The average age was 63.83 ± 5.83 years, including 12 cases of left hemiplegia, 20 cases of right hemiplegia, 8 cases of bilateral hemiplegia, 17 cases of cerebral hemorrhage, and 23 cases of cerebral infarction. In group C, there were 26 males and 14 females; aged 52–74 years; the average age was 65.48 ± 5.29 years old; 14 cases of left hemiplegia, 22 cases of right hemiplegia, and 4 cases of bilateral hemiplegia; 15 cases of cerebral hemorrhage and 25 cases of cerebral infarction. The general data of the three groups were comparable (*P* > 0.05). This study was approved by the hospital ethics committee.

### 2.2. Inclusion Criteria

① All meet the diagnostic criteria of stroke in the “Chinese Guidelines for Early Rehabilitation and Treatment of Stroke” [6] and are accompanied by varying degrees of paralysis; ② All have been diagnosed with stroke by head CT, MRI, and other imaging examinations; ③ Stay in bed ≥3 months; ④ Muscle strength was graded 0–3; ⑤ All volunteered to participate in this study.

### 2.3. Exclusion Criteria

① Patients with other malignant tumors; ② Patients with the worsening condition; ③ Patients with severe orthopedic diseases; ④ Patients with disturbance of consciousness or mental illness; ⑤ Patients with severe organ dysfunction such as heart, liver, and kidney.

### 2.4. Methods

All three groups received drug treatments, such as nourishing cranial nerves and improving cerebral circulation. Group A was given comprehensive outcome-oriented integrated zero-defect nursing combined with respiratory function training, group B was given nursing outcome-oriented integrated zero-defect nursing, and group C was given routine nursing.

### 2.5. Groups C

According to the study manual, group C was given routine medical nursing, regular turning over nursing, limb pressing nursing, diet nursing, and sputum excretion nursing, and learned breathing training such as arm lift breathing training and lip contraction breathing training, according to the study manual.

### 2.6. Group B

① Outcome-oriented, leading indicators of nursing outcomes included psychosocial, community, physical, family, functional, perceived health, and health knowledge and behavior. ② A nursing team should be established with objective management theory. ③ Target incentive scheme. Drafting prevention measures for a lung infection, set up a tiny target in different periods. ④ Prevent aspiration. The supine position should be selected if the patient is in a coma or with blurred consciousness. The patient's head should be tilted to one side, turned over regularly, and a pat on the back for sputum aspiration, clean the patient's respiratory secretions, and keep the patient's respiratory tract unobstructed. Under strict aseptic conditions, sputum aspiration should be carried out gently to avoid infection caused by respiratory mucosal injury. If the patient has difficulty in breathing, the attending physician must be informed in time. If necessary, tracheotomy can be performed. ⑤ DVT prevention. Nurses turned the patient over once every 2 hours and gave massage treatment, from the distal end to the proximal end of the limb, two times a day; instructed the patient to eat a low-salt, low-fat, high-fiber diet and drink more water to ensure unobstructed stool. ⑥ Swallowing function training. Oral exercise training: the tongue depressor was used to stimulate the inside of the cheek, around the lips, and the tongue of the patient, and the patient was instructed to do the actions of extending the tongue, puffing the cheeks, and shrinking the lips, the treatment time was 5 min/time. A disposable frozen long-handled cotton swab was used to dip physiological saline into the patient's soft palate and posterior pharyngeal wall, and the patient was told to do empty swallowing 5 min/per time. Throat lifting exercise: the patient lowered his head slightly, practiced swallowing under the nurse's guidance, and the therapist slightly pushed the patient's throat upward, 5 min/per time. Glottis closure exercise: the patient pressed hard on the desktop and continued to make the “I” sound, 5 min/per time. The above swallowing actions were performed once a day, 20 min/time, 5 d/week, for four consecutive weeks of intervention.

### 2.7. Group A

Based on group B, patients were given breathing function training. ① Patients took semirecumbent positions or sitting positions for deep breathing training. First, patients inhaled deeply through the mouth and nose to make the abdomen heave, then contracted to breathe slowly and evenly through the mouth, and exercised alternately. ② Patients took the sitting or semirecumbent position for glottic function training and inhaled slowly and forcefully through the mouth and nose. The patient was required to use the glottis to exert force, cough forcefully, or make a “P” sound at the end of inspiration. ③ Patients took the sitting or semirecumbent position to shrink the mouth for breathing, use the nose for breathing, shrank the lips to exhale, and exhale as long as possible; the exhalation and the inspiratory ratio was 1 : 2. ④ The patient took the prone position to assist sputum drainage mechanically, and the nurse assisted the patient to turn over and pat his back repeatedly, and pat the bronchus from bottom to top according to the lesion site, two times/day, 20 min/time.

### 2.8. Observation Indicators

① Comparison of the classification of Rosenbek aspiration degree among three groups. Rosenbek aspiration degree classification standard [7] was used for evaluation. When barium agent enters into the laryngeal vestibule but not below the vocal fold, it is leakage, Rosenbek grade is 2∼4; When barium agent enters the laryngeal vestibule and below the vocal fold, it is an aspiration, and Rosenbek grade is 6–8. ② Respiratory function. Before and after the intervention, the pulmonary function detector (Evergrande Electronic Medical) was used to analyze the blood oxygen saturation, arterial blood oxygen partial pressure, and respiratory pressure in the three groups. ③ The water swallowing test (WST) [8] was used to evaluate the swallowing dysfunction of the three groups. Before the test, 30 ml of warm water was prepared, and the drinking conditions of the three groups were observed. The patients were graded from I to V according to their drinking time and the occurrence of choking. Grade I: drink all at once without choking; Grade II: drink more than two times without choking; Grade III: drink all at once with choking; Grade IV: drink more than two times with choking; Class V: challenging to drink, often choking. The higher the grade, the worse the swallowing function. Efficacy evaluation criteria for swallowing function: cure: no swallowing disorder (grade I); markedly effective: the swallowing function was improved, with a gradual improvement of ≥2 grades; effective: the swallowing function was improved, with a gradual improvement of 1 grade; ineffective: no improvement in swallowing function. Total markedly effective rate = cure + markedly effective. ④ Incidence of complications. ⑤ Quality of life. Generic Quality of Life Inventory-74 (GQOLI-74) [9] was used to assess the quality of life of the three groups before and after the intervention. The scale includes four dimensions, including physical function (20 items), psychological function (20 items), social function (20 items), and material life state (10 items), with four factors in each dimension, a total of 16 factors (64 items). The maximum score of each factor is 20 points, and the maximum score of each dimension is 80 points. The higher the score, the better the quality of life.

### 2.9. Statistical Methods

SPSS 20.0 statistical software was used to analyze and process the data. Descriptive statistics were expressed as mean ± SD, and categorical variables were represented as percentages. Continuous variables were evaluated by the Student's *t*-test and categorical by the *χ*^2^ test. The rank data were compared by Wilcoxon rank sum test. *P* < 0.05 indicated statistically significant difference.

## 3. Results

### 3.1. Comparison of Rosenbek Aspiration Degree Classification among the Three Groups

Before treatment, there was no significant difference in Rosenbek aspiration degree classification among the three groups (*P* > 0.05), as shown in Table 1.

After treatment, the Rosenbek aspiration degree classification of the three groups Rosenbek aspiration degree classification of groups A and B were better than that of group C, and the difference was statistically significant (*P* < 0.05), as shown in Table 2.

### 3.2. Comparison of Respiratory Function among the Three Groups

Before treatment, there was no significant difference in blood oxygen saturation, arterial blood oxygen partial pressure, and respiratory pressure among the three groups (*P* > 0.05). After treatment, blood oxygen saturation and arterial partial pressure increased, and respiratory pressure decreased in the three groups; the improvement of respiratory function indexes such as blood oxygen saturation, arterial blood oxygen partial pressure, and respiratory pressure in group A was better than that in groups B and C, and the improvement degree of blood oxygen saturation and arterial blood oxygen partial pressure in group B was better than that in group C, the differences were statistically significant (*P* < 0.05), as shown in Table 3.

### 3.3. Comparison of Swallowing Function among the Three Groups

The swallowing function of groups A and B was better than that of group C; the difference was statistically significant (*P* < 0.05), as shown in Table 4.

### 3.4. Comparison of Complication Rates among the Three Groups

The incidence of complications in groups A and B was lower than that in group C, and the incidence of complications in group A was lower than that in group B, and the differences in the incidence of complications among the three groups were statistically significant (*P* < 0.05), as shown in Table 5.

### 3.5. Comparison of Quality of Life among the Three Groups

Before treatment, there were no significant differences in physical, psychological, social, and material life status among the three groups (*P* > 0.05). After treatment, the scores of psychological function, social function, and material life status of the three groups increased, and each score of groups A and B were higher than that of group C, and each score of group A was higher than that of group B, with statistical significance (*P* < 0.05), as shown in Table 6.

## 4. Discussion

Long-term bedridden patients with stroke are prone to a variety of complications, which seriously affect the quality of life of patients and bring a heavy burden to their families. The nursing outcome-oriented nursing method first determines the nursing goals, makes nursing measures more targeted, is conducive to ensuring the efficient implementation of various nursing measures, and helps to improve the quality of nursing. Integrated zero-defect nursing connects head nurses, doctors, and nurses to fully pay attention to the changes in patient's physical functions and improve nursing efficiency. As the leader of the nursing team, the head nurse is responsible for coordinating and supervising the team members, arranging and coordinating the work of the team members to ensure the smooth completion of the nursing measures. Due to the damage to the cerebral central nervous system in stroke patients, the intracranial pressure continues to increase, which can seriously affect the hypothalamus of patients, increase arterial hypertension, damage pulmonary capillaries, and affect the respiratory function of patients [10–12]. Conventional nursing pays more attention to the patient's essential condition monitoring and respiratory tract management, and the nursing outcome-oriented integrated zero-defect nursing implements specific nursing measures for pulmonary infection, clarifies nursing goals, and improves nursing quality. Long-term bedridden patients with stroke are prone to DVT [13–15], and the nursing outcome-oriented integrated zero-defect nursing also provides targeted prevention and intervention of DVT. Respiratory function training can effectively improve respiratory function but also promote the improvement of swallowing function to a certain extent. The exercise of respiratory muscles in respiratory function training can stimulate the respiratory muscle group, prevent respiratory muscle atrophy and bronchial wall collapse, improve airway clearance ability, promote the coordination of the swallowing muscles and respiratory muscles, and ultimately improve the swallowing function [16, 17]. In this study, group A accepted nursing outcome-oriented integrated zero-defect nursing combined with respiratory function training, group B adopted nursing outcome-oriented integrated zero-defect nursing, and group C was given routine nursing to compare the nursing effects.

In this study, Rosenbek aspiration degree classification in groups A and B was superior to that in group C, indicating that nursing outcome-oriented integrated zero-defect nursing can effectively improve aspiration in long-term bedridden patients with stroke. Due to uncoordinated breathing, patients after stroke tend to inhale during swallowing, resulting in aspiration and choking. The nursing outcome-oriented integrated zero-defect nursing has targeted aspiration prevention and effectively reduced aspiration through sputum aspiration, regular turning over, and other measures. In addition, the results of this study showed that after the intervention, the improvement degree of respiratory function indexes such as blood oxygen saturation, arterial partial pressure, and respiratory pressure in group A was better than that in groups B and C, and the improvement degree of respiratory function indexes such as blood oxygen saturation and arterial partial pressure in group B was better than that in group C. The effective rate of swallowing function in groups A and B was higher than that in group C, indicating that the nursing outcome-oriented integrated zero-defect nursing combined with respiratory function training can effectively improve patients' respiratory and swallowing function. The nursing outcome-oriented integrated zero-defect nursing includes swallowing function training, which can fully exercise the swallowing muscle through mouth movement, swallowing action, and glottis closing exercise, and finally improve swallowing function effectively, among which glottis exercise is also helpful to improve respiratory function. Respiratory function training promotes the accumulation of sputum in the large airway to the trachea and larynx, glottis training can prevent the atrophy of respiratory muscles, improve alveolar ventilation, and promote the removal of respiratory secretions, and mouth contraction training can also help improve the muscle strength of mouth and lip and improve swallowing function [18–20]. Therefore, the nursing outcome-oriented integrated zero-defect nursing combined with respiratory function training has a better effect on improving patients' respiratory function and swallowing function. The complication rate of groups A and B was lower than that of group C, and that of group A was lower than that of group B. In this study, DVT, pulmonary infection, and aspiration were the main common complications of long-term bedridden patients with stroke. The nursing outcome-oriented integrated zero-defect nursing includes nursing measures for pulmonary infection, and DVT is prevented from regular turning over, massage, appropriate diet, and other aspects. Swallowing function training and preventing aspiration can effectively improve respiratory function and reduce the incidence of pulmonary infection. After treatment, the scores of psychological function, social function, and material life status of the three groups increased, and each score of groups A and B were higher than that of group C, while each score of group A was higher than that of group B, and the differences were statistically significant (*P* < 0.05). The results showed that the nursing outcome-oriented integrated zero-defect nursing combined with respiratory function training could effectively improve the quality of life of long-term bedridden patients with stroke, and the improvement of the quality of life was closely related to the improvement of their respiratory quality and swallowing function. The patients' respiratory function, swallowing function, and complication rate were significantly improved through the nursing outcome-oriented integrated zero-defect nursing combined with respiratory function training, so patients' quality of life was significantly improved.

In conclusion, the nursing outcome-oriented integrated zero-defect nursing combined with respiratory function training can effectively improve the respiratory function and swallowing function of patients with stroke, reduce the incidence of complications, and improve the quality of life of patients, which has clinical application value.

## Figures and Tables

**Table 1:** Comparison of Rosenbek aspiration degree classification among the three groups before treatment [case (%)].

Group	1	2	3	4	5	6	7	8
Group A (*n* = 40)	4 (10.00)	6 (15.00)	5 (12.50)	6 (15.00)	4 (10.00)	5 (12.50)	4 (10.00)	6 (15.00)
Group B (*n* = 40)	3 (7.50)	5 (12.50)	6 (15.00)	7 (17.50)	5 (12.50)	5 (12.50)	5 (12.50)	4 (10.00)
Group C (*n* = 40)	4 (10.00)	5 (12.50)	5 (12.50)	5 (12.50)	6 (15.00)	6 (15.00)	4 (10.00)	5 (12.50)
z value	0.018							
*P* value	0.991							

*Note. b* indicated *P* < 0.05 when compared with group B; *c* indicated *P* < 0.05 with group C.

**Table 2:** Comparison of Rosenbek aspiration degree classification among the three groups after treatment [case (%)].

Group	1	2	3	4	5	6	7	8
Group A (*n* = 40)	10 (25.00)^c^	10 (25.00)^c^	9 (22.50)^c^	6 (15.00)^c^	2 (5.00)^c^	1 (2.50)^c^	1 (2.50)^c^	1 (2.50)^c^
Group B (*n* = 40)	9 (22.50)^c^	9 (22.50)^c^	8 (20.00)^c^	5 (12.50)^c^	4 (10.00)^c^	3 (7.50)^c^	2 (5.00)^c^	1 (2.50)^c^
Group C (*n* = 40)	5 (12.50)	5 (12.50)	5 (12.50)	5 (12.50)	7 (17.50)	7 (17.50)	3 (7.50)	3 (7.50)
*χ * ^*2*^ value	11.175							
*P* value	0.004							

*Note. b* indicated *P* < 0.05 when compared with group B; *c* indicated *P* < 0.05 with group C.

**Table 3:** Comparison of respiratory function among the three groups (‾*x* ± *s*).

Group	Oxygen saturation (%)		Arterial partial pressure (mmHg)		Respiratory function (cm H_2_O)	
	Before treatment	After treatment	Before treatment	After treatment	Before treatment	After treatment
Group A (*n* = 40)	89.94 ± 2.36	98.32 ± 2.10^abc^	87.77 ± 2.26	98.69 ± 1.89^abc^	26.93 ± 1.45	18.58 ± 1.37^abc^
Group B (*n* = 40)	90.85 ± 2.04	95.70 ± 2.84^ac^	87.63 ± 1.28	93.75 ± 1.43^ac^	26.62 ± 1.55	23.71 ± 2.45^a^
Group C (*n* = 40)	90.87 ± 2.43	92.57 ± 1.74^a^	86.81 ± 1.98	91.59 ± 1.65^a^	26.73 ± 1.84	24.68 ± 2.08^a^
*F* value	2.157	64.113	3.017	190.423	0.382	105.857
*P* value	0.120	<0.001	0.053	<0.001	0.683	<0.001

*Note.*an indicated *P* < 0.05 when compared with the same group before intervention; *b* indicated *P* < 0.05 when compared with group B; *c* indicated *P* < 0.05 when compared with group C.

**Table 4:** Comparison of swallowing function among the three groups [cases (%)].

Group	Cure	Markedly effective	Effective	Ineffective	Total effective rate
Group A (*n* = 40)	13 (32.50)	21 (52.50)	4 (10.00)	2 (5.00)	34 (85.00)^c^
Group B (*n* = 40)	10 (25.00)	18 (45.00)	5 (12.50)	7 (17.50)	28 (70.00)^c^
Group C (*n* = 40)	6 (15.00)	8 (20.00)	15 (37.50)	11 (27.50)	14 (35.00)
*χ * ^*2*^ value					22.679
*P* value					<0.001

*Note. b* indicated *P* < 0.05 when compared with group B; *c* indicated *P* < 0.05 with group C.

**Table 5:** Comparison of the incidence of complications among the three groups [cases (%)].

Group	DVT	Pulmonary infection	Aspiration	Total complication rate
Group A (*n* = 40)	1 (2.50)	4 (10.00)	1 (2.50)	6 (15.00)^bc^
Group B (*n* = 40)	3 (7.50)	9 (22.50)	2 (5.00)	14 (35.00)^c^
Group C (*n* = 40)	10 (25.00)	15 (37.50)	12 (30.00)	37 (92.50)
*χ * ^*2*^ value				51.930
*P* value				<0.001

*Note. b* indicated *P* < 0.05 when compared with group B; *c* indicated *P* < 0.05 with group C.

**Table 6:** Comparison of quality of life among the three groups (‾*x* ± *s*).

Group	Physical function		Psychological function		Social function		Material life status	
	Before treatment	After treatment	Before treatment	After treatment	Before treatment	After treatment	Before treatment	After treatment
Group A (*n* = 40)	42.50 ± 8.91	45.13 ± 4.99	31.25 ± 6.00	65.03 ± 7.60^abc^	34.25 ± 6.74	71.38 ± 6.17^abc^	22.23 ± 4.12	45.28 ± 3.97^abc^
Group B (*n* = 40)	42.90 ± 4.49	44.68 ± 4.48	32.33 ± 4.52	59.58 ± 5.91^ac^	33.58 ± 5.27	65.85 ± 6.44^ac^	22.13 ± 3.27	38.20 ± 3.83^ac^
Group C (*n* = 40)	40.00 ± 6.84	44.63 ± 5.16^a^	32.20 ± 3.65	53.78 ± 6.41^a^	33.18 ± 6.41	60.83 ± 6.16^a^	21.48 ± 2.04	29.80 ± 3.29^a^
*F* value	2.026	0.127	0.594	28.389	0.310	28.478	0.626	174.587
*P* value	0.136	0.881	0.554	<0.001	0.734	<0.001	0.536	<0.001

*Note.*an indicated *P* < 0.05 when compared with the same group before intervention; *b* indicated *P* < 0.05 when compared with group B; *c* indicated *P* < 0.05 when compared with group C.

## Data Availability

The labeled dataset used to support the findings of this study are available from the corresponding author upon request.
